The article "Digital transformation, industrial structure change, and economic growth motivation: An empirical analysis based on manufacturing industry in Yangtze River Delta" was retracted in 2025. Reasons: unreliable results or conclusions; concerns about the peer review; concerns about the authorship; concerns about the article.

# Digital transformation, industrial structure change, and economic growth motivation: An empirical analysis based on manufacturing industry in Yangtze River Delta

**DOI:** 10.1371/journal.pone.0284803

**Published:** 2023-05-17

**Authors:** Xuefeng Zheng, Xiufan Zhang, Decheng Fan

**Affiliations:** 1 School of Economics and Management, Harbin Engineering University, Harbin, China; 2 School of Management, Heilongjiang University of Science and Technology, Harbin, China; 3 School of Economics and Management, Zhejiang Sci-Tech University, Hangzhou, China; Shenzhen University, CHINA

## Abstract

China is in a critical stage of economic growth mode transformation. The digital transformation of the manufacturing industry may create new impetus and new models for economic growth. Taking the manufacturing industry of 25 prefecture-level cities in the Yangtze River Delta region as the research object, we explore the digital transformation process of the manufacturing industry and verifies its theoretical mechanism of promoting economic growth through the industrial structure. A panel model based on the improved Feder two-sector model and a multiple mediating effect model are established to explore the dynamic mechanism of manufacturing digital transformation to promote economic growth through industrial restructuring. The results show that the digital transformation of the manufacturing industry in the Yangtze River Delta region of China is relatively high, and the speed of digital transformation has been accelerating in recent years. The digital transformation of the manufacturing industry can promote the change in industrial structure and form a new driving force for economic growth. The key is to improve the level of industrial structure and extend the length of the industrial chain. Based on these, we propose measures to promote the transformation and upgrading of industrial structure for the sustainable development of China’s economy.

## 1. Introduction

Digital transformation is an innovative process based on the combination of digital technologies such as information computing, communication, and connectivity to trigger entity attributes. With the rapid development of the digital economy, digital technology represented by the Internet and big data is deeply integrated with the manufacturing industry. The development of the manufacturing industry takes digital platforms as the medium, which greatly changes the production and organization management mode of enterprises. In recent years, China has issued a series of relevant policies to promote digital transformation, and the manufacturing industry has accelerated the process of digital transformation. As of October 2021, China has established more than 130 industrial Internet platforms and developed 80 million manufacturing digital devices, which has become an important driving force for improving production and management efficiency and optimizing industrial structure. At present, the existing research is mainly from the following perspectives; first, digital technology is conducive to improving production efficiency. Introducing digital technologies such as the Internet and artificial intelligence into production, management, business, and other links and chains, can enhance the information collection and large-scale interaction capabilities of the production side, drive efficient and connected production methods, and improve the total factor productivity of enterprises. Vacchi et al. pointed out that the development of the digital economy can promote the optimization and upgrading of the production mode of the manufacturing industry, and profoundly affect the digital transformation of the manufacturing industry from the demand side, production side, and management side [1]. Second, digital transformation is conducive to business expansion, helping enterprises achieve value creation in the production process and increase procurement channels [2]. However, some scholars suggest that although the current momentum of development of China’s digital economy is good, the classification between provinces is obvious [3]. The problem of the ’’digital divide’’ is still serious, and the digital transformation of enterprises still needs a period of adaptation time [4, 5]. Third, digital transformation reduces transaction costs through information resource integration and forms competitive advantages in the process of organizational management [6]. At the same time, conflicts between old and new resources and systems may arise in the process of digital transformation, which brings uncertainty to enterprise development [7, 8]. Digital transformation faces high energy consumption problems. Fourth, digital technology promotes industrial integration, thereby further expanding the value chain [9, 10]. The digital economy has promoted the gradual integration of the manufacturing industry and the service industry, making the manufacturing industry tend to be service-oriented and becoming the director of the integrated development and upgrading of the manufacturing industry.

The article "Digital transformation, industrial structure change, and economic growth motivation: An empirical analysis based on manufacturing industry in Yangtze River Delta" was retracted in 2025. Reasons: unreliable results or conclusions; concerns about the peer review; concerns about the authorship; concerns about the article.

However, few literature examine the driving force of digital transformation on economic growth from the perspective of the industry. Therefore, we take the manufacturing industry in the Yangtze River Delta region as the research object, introduce the industrial perspective, conduct in-depth research on the impact mechanism of digital transformation on economic growth, and form the following path: ’manufacturing digitization→industrial restructuring→economic growth’. Second, from the perspective of industrial structure, analyze the differential impact of manufacturing digitization. In contrast, the digitalization of the manufacturing industry has a more significant impact on the upgrading of industrial structure and the length of the industrial chain, and the mediating effect of the two on economic growth is more significant. We reveal the internal mechanism of the digital transformation of the manufacturing industry to promote economic growth. The research explains the internal driving force of digital transformation in the manufacturing industry to promote economic growth based on dynamic capability, organizational structure, resource investment, and business process from a deeper perspective.

## 2. Literature review

### 2.1. Manufacturing digitization and economic growth

The cognitive framework of mainstream economics usually discusses the constraints of economic growth from demand and supply and divides economic growth into demand-driven growth and supply-driven growth. Digital transformation of the manufacturing industry makes the industrial structure, by adjusting the supply side structure to provide new impetus for economic growth. Wang Yiming conducted an in-depth study on the impact of digital development on the upgrading of industrial structures in 30 provinces of China. He believes that, on the one hand, as a new factor of production, data promotes the development of enterprises to the high-end link while expanding the scale of production, transforming and upgrading traditional processes, and opening up markets, thus expanding the external space of economic growth, strengthening its role in economic growth and forming strong traction [11]. The coronavirus epidemic has had a major impact on economic development [12–14]. Therefore, manufacturing digitalization can effectively promote the flow of resources and factors, integrate multi-agent production efficiency, and improve economic vitality.

As the traditional competitive advantage of the manufacturing industry gradually weakens, it brings severe challenges to the sustainability of the economic growth mode and dynamic mechanism [15, 16]. The competitive advantage of the manufacturing industry is mainly to reduce production costs and form a competitive advantage by forming economies of scale to reduce prices and increase production capacity [17]. However, in recent years, with the rapid increase of labor, land, and environmental costs, the advantages brought by low-cost strategies have gradually weakened. Economic growth needs to be adjusted to a dynamic mechanism driven by technological innovation and production efficiency [18, 19]. In recent years, scholars have continuously proposed that capital input should dominate economic growth. Resource allocation and industrial structure can play an important role in economic growth [20–22]. According to the "Manufacturing Quality Management Digital Implementation Guide (Trial)", data is an important factor of production, which is different from traditional factors of production such as labor and land. It has the attributes of sharing and unlimited supply, which can support enterprise decision-making, realize the coordinated development of factors, and vigorously promote technological innovation.

The article "Digital transformation, industrial structure change, and economic growth motivation: An empirical analysis based on manufacturing industry in Yangtze River Delta" was retracted in 2025. Reasons: unreliable results or conclusions; concerns about the peer review; concerns about the authorship; concerns about the article.

During the ’14th Five-Year’ period, China has made every effort to speed up the all-round and full-chain transformation of manufacturing enterprises by digital technology. The attributes of digitalization determine that it has a positive effect of amplification, superposition, and multiplication on economic growth. China has put forward the development goal of increasing the added value of digital core industries to 10% of China’s GDP by 2025. Therefore, digitization can stimulate technological innovation, promote efficiency improvement, and optimize resource allocation to build a market system and external environment driven by innovation and efficiency, which is an important production factor for economic growth.

### 2.2. Manufacturing digitalization and industrial structure upgrading

Manufacturing digitalization can improve the dynamic development efficiency of the industry and promote the integrated development of the industrial chain, thus forming an important engine and driving force for economic growth more effectively [23, 24]. With the accelerated development of manufacturing digitalization, the industrial structure has significantly increased the speed of capital accumulation, which in turn has led to the economic growth led by the input of production factors such as technology, data, and capital [25, 26].

Digital technology leads enterprises to formulate new development strategies to adapt to the highly competitive market environment and promote the transformation and upgrading of industrial structure [27, 28]. Xue et al. conducted an empirical study on the panel data of 30 provinces in China to analyze the far-reaching impact of the digital economy on the industrial structure. He believed that digital technology could improve the efficiency of production factors such as technology flow, capital flow, and talent flow in the whole process of industrial production [29]. On the one hand, data is a new factor of production, which can achieve the coincidence of factors of production, change the original resources and production patterns, promote intelligent manufacturing, and realize the reduction of production costs. On the other hand, digital technology improves the operation mode, realizes multi-system interaction, and realizes the upgrading of industrial structure, making intelligent manufacturing gradually become the mainstream trend of manufacturing development [30]. With the continuous penetration of the breadth and depth of the Internet, a new digital production mode can be further created. Manufacturing enterprises carry out remote operation and monitoring information services to derive new ways of the division of labor and cooperation, changing the traditional manufacturing development system, which can greatly improve production efficiency.

The article "Digital transformation, industrial structure change, and economic growth motivation: An empirical analysis based on manufacturing industry in Yangtze River Delta" was retracted in 2025. Reasons: unreliable results or conclusions; concerns about the peer review; concerns about the authorship; concerns about the article.

### 2.3. Manufacturing digitalization and industrial structure rationalization

The manufacturing digitalization accelerates the flow of production factors and realizes the sharing of information and technology, which leads to the transformation of production mode, technology, and mode, promotes the formation of a more active flow and interaction of factors among industries, and gradually adjusts the industrial structure towards the rational development of technology, structure, quality, and resources [31, 32]. Tong et al. analyzed the impact of digital economy development on industrial structure based on panel data of 30 provinces in China and found that digital economy can drive industrial structure to rationalize development [33]. From the perspective of the labor force, the improvement of digital technology and the construction of digital platforms will greatly increase the production cost of enterprises, but it would promote the improvement of staff quality and make the industrial structure tend to be rationalized [34, 35]. Fossen and Sorgner conducted an in-depth study on the impact of digital transformation on production methods. The results show that the process of digital transformation, will lead to the upgrading and transformation of key production factors of enterprises, and promote enterprises to gradually change their production methods, thus promoting the rationalization of industrial structure [36]. Navarro and Garay empirically tested the mechanism of digital transformation and industrial structure, arguing that digital transformation can positively affect the rationalization of industrial structure [37]. Through the establishment of a comprehensive and efficient most modern information management system, the manufacturing industry promotes the information exchange and efficient integration of information between different departments of the enterprise. Manufacturing enterprises run through the application of digital technology in product design, part production, product assembly, product circulation, marketing operation, after-sales service, and other links, which has an important impact on the production and management decision-making of enterprises [38, 39]. It helps to provide a good basis for decision-making ability and change the manufacturing production mode. In the business process, digital technologies such as big data analysis, artificial intelligence, and the Internet of Things, as well as data platforms and business platforms, are used to improve the refined management level of enterprises.

The article "Digital transformation, industrial structure change, and economic growth motivation: An empirical analysis based on manufacturing industry in Yangtze River Delta" was retracted in 2025. Reasons: unreliable results or conclusions; concerns about the peer review; concerns about the authorship; concerns about the article.

### 2.4. Manufacturing digitalization and industrial integration

The integration and penetration of the manufacturing industry and information industry make technological innovation and resource sharing emerge, interact among enterprises, promote the integration of related industries, and bring new impetus to development [40, 41]. The data platform enables information sharing between different industries, and the form of cross-industry integration development is emerging, driving the upgrading of production factors, and thus promoting the improvement of production efficiency. Liu et al. conducted an empirical study on the spatial panel data of 30 provinces in China and verified the spatial effect of digital transformation on industrial integration [42]. The manufacturing industry, which is gradually integrated with informatization and servitization, uses information networks to continuously expand the production mode, to realize intelligent production and manufacturing. The intelligent production mode is the most direct embodiment of the integration of industrialization and informatization [43, 44]. Manufacturing enterprises can use the information system to change the original large-scale, inefficient and repetitive flow-line operation so that the production mode tends to be multi-type, high-quality, and personalized. The program effectively changes the original production level and management mode of the manufacturing industry.

### 2.5. Manufacturing digitalization and extension of the industrial chain

China vigorously promotes the digital development of the manufacturing industry, aiming at improving the intelligent development of key links in the industrial chain, improving productivity, and improving the supply chain system of the manufacturing industry. By using modern digital technologies and equipment such as big data analysis, virtual reality, blockchain, data crawler, etc., real-time statistical collection and analysis of operational information are completed to improve the sensitivity of supply and demand side response [44]. Digitization and related technologies play an important role in the extension and management innovation of the industrial chain. This is not only reflected in the intelligent development of the industry but also reflected in the industrial chain between the upstream and downstream data analysis and decision-making. On the one hand, by using new equipment such as sensors and wireless technology, the data and information generated in the production process are fully captured, and form an intelligent network among organizations [45]. While reducing production costs, digital technology effectively improves the reliability of equipment, and monitors and analyzes the development process of the industrial chain, enabling real-time optimization in the production process [46]. Through the data collected by the whole channel, the extension of the industrial chain is realized, and the guidance operation is more referenced.

The article "Digital transformation, industrial structure change, and economic growth motivation: An empirical analysis based on manufacturing industry in Yangtze River Delta" was retracted in 2025. Reasons: unreliable results or conclusions; concerns about the peer review; concerns about the authorship; concerns about the article.

## 3. Experimental

### 3.1. Research object introduction

The Yangtze River Delta Urban Agglomeration (abbreviation: Yangtze River Delta Urban Agglomeration) is located in the alluvial plain before the Yangtze River enters the sea. According to the "Yangtze River Delta Urban Agglomeration Development Plan" approved by the State Council, the Yangtze River Delta Urban Agglomeration includes: Shanghai, Nanjing, Wuxi, Changzhou in Jiangsu Province etc., Hangzhou, Ningbo, Jiaxing, etc. in Zhejiang Province, Hefei, Wuhu, Ma’anshan and other 25 cities in Anhui Province. The Yangtze River Delta urban agglomeration is an important intersection between the "Belt and Road" and the Yangtze River Economic Belt, and is an important modern service industry and advanced manufacturing center in the world. Accelerate the promotion of cross-industry integration, focus on the development of high value-added industries, high value-added links and the headquarters economy, accelerate the cultivation of new competitive advantages centered on technology, brand, quality and service, and create a number of advanced manufacturing industries that are at the forefront of international scale and level Cluster to form a modern industrial system dominated by the service economy and supported by intelligent manufacturing.

### 3.2. Evaluation index selection

Digital transformation enables manufacturing to form multi-level complex systems and behaviors. For the measurement of the digital transformation level of the manufacturing industry, scholars have proposed information development indicators [47, 48], Internet development indicators [49], and digital transaction indicators. Fleischer analyzed the evolution of digital transformation from the perspectives of the digital platform [50]. Digital transformation enables the manufacturing industry to effectively reduce the cost of collecting, storing, and processing various types of information by building a digital platform. By reconstructing dynamic capabilities, the manufacturing industry introduces intelligent equipment, creating new ways of value creation, adjusting business processes, and simplifying the production process [51–53]. On the other hand, some scholars believe that in the highly changing digital environment, enterprises reshape the digital development vision, build digital transformation strategy, and develop dynamic capabilities, to guide the deep application in the whole process and multi-link of R&D, production, organization, and management. Some scholars have evaluated the digital transformation from the dimensions of value, elements, and ability, but the research on manufacturing enterprises needs to be further refined. Based on this, the key elements of digital transformation in the manufacturing industry are summarized, and the level of digital transformation is measured from three aspects: dynamic capability, digital platform, and organizational system.

The article "Digital transformation, industrial structure change, and economic growth motivation: An empirical analysis based on manufacturing industry in Yangtze River Delta" was retracted in 2025. Reasons: unreliable results or conclusions; concerns about the peer review; concerns about the authorship; concerns about the article.

### 3.3. Digital capability transformation

Dynamic capability is an important theory to analyze the manufacturing industry adapting to the digital transformation environment [54]. Dynamic capabilities mainly include environmental awareness capabilities, information acquisition capabilities, resource transformation capabilities, and multi-dimensional integration capabilities, thereby improving management processes, optimizing organizational management, and improving adaptability to digital technologies [55, 56].

Ability to perceive the environment: this indicator helps manufacturing industries use digital technology to discover and create opportunities to digitally ’empower’ through scanning, evaluation, calibration, and analytical actions [57]. Scanning ability reflects the ability of enterprises to collect and filter internal and external information. Evaluation ability reflects the ability of enterprises to learn and evaluate potential opportunities; calibration capability refers to the ability of enterprises to clarify future actions and strategies in the process of digital transformation. In a highly competitive market, manufacturing understands market demand and expands customer preferences by analyzing big data [58].

The key ability of manufacturing enterprises through data mining, scheme selection, and information operation in the process of digital transformation, including design ability, selection ability, and operation ability [59]. Design capability refers to the ability of enterprises to plan and design new structures by mining, collecting, and recycling data. Selection ability refers to the ability of enterprises to choose potential solutions through digital technology, including suppliers, services, and business models [60]. Operational capability is the ability to form new products, processes, or services through big data operations, investment, and development [61].

The article "Digital transformation, industrial structure change, and economic growth motivation: An empirical analysis based on manufacturing industry in Yangtze River Delta" was retracted in 2025. Reasons: unreliable results or conclusions; concerns about the peer review; concerns about the authorship; concerns about the article.

Manufacturing enterprises should rely on rich data to form resource advantages and produce a leverage effect [62]. Arranging digital resources, enabling digital ecology to realize value creation, thus providing important support for the future development of enterprises [63]. Specifically, the resource transformation ability of manufacturing enterprises includes release ability, reset ability, and creative ability. Releasing capacity is the ability of enterprises to reorganize resources for digital strategies in the face of knowledge transfer, resource adjustment, and information absorption to organize internal and external resources, thereby reducing dependence on inherent paths, developing external capital, and supplementing existing resources [64]. Reconfiguration capability refers to the ability of enterprises to reconfigure assets to improve their digital transformation and explore new forms of development through digital platforms [65].

Multidimensional integration capability helps companies reduce technology transaction costs through data platforms, participate in ecosystems by integrating digital technologies provided to multiple parties, and actively adapt to the strategic goals of digital transformation.

### 3.4. Digital platform transformation

The digital platform is a carrier for communicating external resources and internal collaborative decision-making to achieve value co-creation. The digital platform is an important carrier of data to support user aggregation, information interaction, and value exploration [66]. The distributed character of the digital platform makes it merge with organizational systems and digital technology to derive new development power [67].

Platform architecture represents the interactive innovation and continuous optimization of organizational structure. Digital components are introduced into the structural design of the platform to improve the original attributes, focus on data integration, and build the platform around the production and consumption, technological innovation, energy, and environmental protection of the manufacturing industry [68]. The digital ecology of efficient coordination, complementary advantages, and mutual benefit enables manufacturing enterprises to continuously meet the needs of economic growth.

The article "Digital transformation, industrial structure change, and economic growth motivation: An empirical analysis based on manufacturing industry in Yangtze River Delta" was retracted in 2025. Reasons: unreliable results or conclusions; concerns about the peer review; concerns about the authorship; concerns about the article.

The collaborative integration represents the efficiency of resource allocation in manufacturing enterprises, realize the transformation of resource control into efficient use of resources, and externalize internal advantages into information interaction [69]. Collaborative integration aims to achieve wide-area business development, connectivity, and integration, and enhance the scope of adaptation and adaptability of manufacturing enterprises. Digital collaborative integration enables enterprises to expand the coverage of multiple fields and subjects, and enhance the breadth of interaction between enterprises and markets [70].

Business and scenario-driven is the simulation of business and scenario-driven in the process of platform construction. As the platform’s driving force for business continues to increase, the popularity of enterprises has increased rapidly, helping to form unique new technology products [71]. At the same time, the scene-driven improves the ability of enterprises to modify the environment and enhances the influence and driving force of manufacturing enterprises on the market environment through platform construction.

Therefore, the digital platform can improve the operation mode of enterprises, realize automatic management and efficient production, and adapt to the highly competitive market environment [72]. The digital platform is a production and operation mode that uses the new generation of information technologies such as the Internet, big data, cloud computing and artificial intelligence to build a digital platform, data management, data operation, data decision-making and innovation [73]. In essence, its core is data, including data acquisition, data storage, data utilization, data prediction and data security maintenance. Taking industrial software and embedded system software as the carrier, the deep integration of manufacturing industry and IT industry is realized through technological transformation.

### 3.5. Digital applications

In the process of digital transformation of manufacturing enterprises, the organizational system has gradually changed, injecting evolutionary power into the development of enterprises and the transformation of industrial structure [74]. The organizational system reform brought by digital transformation includes organization model construction, cross-business process construction, and weakening organization conflict [75]. The organization establishes a more precise strategic framework in the process of digital transformation to better play the function of information functional departments. The whole life cycle management of the process is realized through a digital information system [76]. The digital transformation of a business process can realize the high-level evolution of knowledge and information, promote manufacturing enterprises to form digital interaction in key areas, and promote the integration of the organization management and community information system [77].

The article "Digital transformation, industrial structure change, and economic growth motivation: An empirical analysis based on manufacturing industry in Yangtze River Delta" was retracted in 2025. Reasons: unreliable results or conclusions; concerns about the peer review; concerns about the authorship; concerns about the article.

Resolving the conflict of organizational systems in the process of digital transformation requires weakening the differences in organizational culture and development strategies at the implementation level of the organization. Through the design of a digital interface to maintain the consistency of the rules of behavior on both sides of the organization, establish an effective association structure. In the multi-level development of the organization, the linkages between individual and organizational levels of development are coordinated and risk resilience is formed to enable enterprises to effectively resolve risks in the face of digital transformation challenges.

The digital transformation of manufacturing enterprises penetrates multiple links of the value chain, realizes value co-creation through resource allocation and planning, improves production efficiency, helps enterprises optimize production processes, and improves economic and ecological benefits [78]. Digital benefit transformation refers to the economic and ecological benefits created by digital transformation to enterprises, that is, to improve the economic benefits of enterprises while better assuming the social responsibility of enterprises. In essence, the core of digital benefit transformation lies in value [79]. Digital industrialization, industrial transformation and ecological environment, the digital benefits are divided into economic benefits and ecological benefits, and the ecological benefits are considered from energy and environment [80].

### 3.6. Expert selection of evaluation index based on Delphi method

Experts will be selected for the evaluation index system of digital innovation ability initially constructed above. We use the Delphi method for selection and decision-making. This study strictly follows the investigation process, and professionals express their views in an anonymous manner to ensure that they are independent and free to judge, and there is no cross-relationship. Using the Delphi method, the established evaluations were summarized twice. During the research period, we communicate closely with various professionals, and actively collect expert correction suggestions, and integrate the opinions of various professions to form two stages of evaluation indicators. After collecting a large number of professional research results, a new evaluation index of enterprise digital innovation ability is obtained, and the index is predicted and analyzed by two experts, to modify the evaluation results and make the evaluation results more scientific.

1. Constructing expert consultation indicators

The evaluation index of digital innovation ability initially constructed above is distributed to various experts in the form of questionnaires. The scope of expert selection includes: 6 experts in the field of digital technology, 8 professional and technical personnel, and 6 executives of A company who were randomly selected. Experts vote on the initial evaluation index system of digital innovation ability, so as to select the evaluation index of digital innovation ability. The evaluation index system of the degree of digital transformation of manufacturing industry is shown in Table 1.

The article "Digital transformation, industrial structure change, and economic growth motivation: An empirical analysis based on manufacturing industry in Yangtze River Delta" was retracted in 2025. Reasons: unreliable results or conclusions; concerns about the peer review; concerns about the authorship; concerns about the article.

**Table 1:** Evaluation index system of digital transformation of the manufacturing industry.

First-level indicators	Second-level indicators	Indicator measure	Unit
Digital Capability Transformation (A)	R&D intensity A1	R&D expenditure internal expenditure / main business income	%
	Product innovation ability A2	New product sales revenue / main business income	%
	Digital talent reserve A3	Number of employees in software and information technology service industry	Thousand people
	Effective number of invention patents A4	The number of invention patents within the validity period of the reporting year in the region	Piece
Digital platform transformation (*B*)	Digital equipment investment B1	Fixed asset investment in software and information technology services	RMB 100 million
	Communication and network coverage capabilities B2	Number of Internet broadband access ports	Ten thousand
	Data processing and operation ability B3	Information systems integration services revenue, data processing and operations services revenue	Ten thousand yuan
	Digital software application B4	The sum of software product income, information technology service income and embedded system software income.	Ten thousand yuan
	Digital security construction ability B5	Information security software revenue	Ten thousand yuan
Digital Applications(*C*)	E-commerce development level C1	Enterprise average e-commerce turnover	Ten thousand yuan
	the electronic information manufacturing industry digital development status C2	Electronic information manufacturing industry operating income as a share of GDP	%
	Information transmission, computer services and software industry investment scale C3	Information transmission, computer services and software industry Fixed investment / fixed asset investment	%
	Big data industrial application index C4	Big data industrial application index	

The article "Digital transformation, industrial structure change, and economic growth motivation: An empirical analysis based on manufacturing industry in Yangtze River Delta" was retracted in 2025. Reasons: unreliable results or conclusions; concerns about the peer review; concerns about the authorship; concerns about the article.

### 3.7. Composition and weight calculation of index system

Considering the dynamic nature of the evaluation index of digital transformation of manufacturing industry constructed in this study, the TOPSI method is used (Hwang & Yoon, 1987).

2. Entropy method to determine the index weight

The first step is to construct the original matrix with *m* objects and *n* indexes.

In the second step, in order to avoid the error in the calculation of different dimensions, the original matrix is homogenized and normalized to obtain the standard matrix.


$$V={\left[v_{ij}\right]}_{m\times n}$$

The third step is to use the entropy weight method to calculate the weight *w* of each index.


$$w_{j}=\frac{1-e_{j}}{n-\sum_{j=1}^{n}e_{j}}$$

Where, $e_{j}=-\frac{1}{\ln\;m}\sum_{i=1}^{m}p_{ij}\ln\;p_{ij}$, $p_{ij}=v_{ij}/\sum_{i=1}^{m}v_{ij}$

Determine the positive ideal solution and negative ideal solution:

$$p^{+}=(v_{1}^{+},v_{2}^{+},\ldots ,v_{j}^{+}),i=1,2,\ldots ,p;j=1,2,\ldots ,q$$

$$v_{j}^{+}=\{(\max\;v_{ij}|j\in J_{1}),(\min\;v_{ij}|j\in J_{2}),i=1,2,\ldots ,p\}\;p^{-}=(v_{1}^{-},v_{2}^{-},\ldots ,v_{j}^{-}),i=1,2,\ldots ,p;j=1,2,\ldots ,q$$

$$p^{-}=(v_{1}^{-},v_{2}^{-},\ldots ,v_{j}^{-}),i=1,2,\ldots ,p;j=1,2,\ldots ,q\;v_{j}^{-}=\{(\min\;v_{ij}|j\in J_{1}),(\max\;v_{ij}|j\in J_{2}),i=1,2,\ldots ,p\}$$

*J*_*1*_ is the benefit index set and *J*_*2*_ is the cost index set. Calculate the distance from each sample to positive and negative ideal points ($d_{i}^{*}$), ($d_{i}^{-}$)

$$d_{i}^{*}=\sqrt{\sum_{j=1}^{q}{\left(v_{ij}-v_{j}^{+}\right)}^{2}},i=1,2,\ldots ,p;j=1,2,\ldots ,q$$

$$d_{i}^{-}=\sqrt{\sum_{j=1}^{q}{\left(v_{ij}-v_{j}^{-}\right)}^{2}},i=1,2,\ldots ,p;j=1,2,\ldots ,q$$

Calculate the progress of the index *C*(*s*_*i*_)

$$C_{i}^{*}=\frac{d_{i}^{-}}{d_{i}^{-}+d_{i}^{+}},i=1,2,\ldots ,p$$

Relevant specific data sets can be accessed through direct hyperlinks. Others will be able to access or request this data in the same way as the author, who does not have any special access or request privileges that others will not have.

Data sources: China Statistical Yearbook: http://www.stats.gov.cn/sj/ndsj/:

China Digital Economy Development Report: https://www.xdyanbao.com/doc/ivfqexmap4;

China Big Data Regional Development Level Assessment White Paper:

http://www.199it.com/archives/tag/%E8%B5%9B%E8%BF%AA%E6%99%BA%E5%BA%93

China High-tech Industry Statistical Yearbook’:

https://www.yearbookchina.com/navibooklist-n3020013209-1.html

https://jw.cnki.net/KNavi/yearbook/Detail/WWBY/YBVCX

China ’s new infrastructure competitiveness index white paper:

https://www.sgpjbg.com/luodi/240931.html?tg=1&plan=%e8%a1%8c%e4%b8%9a%e6%8a%a5%e5%91%8a18-%e8%bf%81%e7%a7%bb-%e7%99%bd%e7%9a%ae%e4%b9%a6&keyword360=%e4%b8%ad%e5%9b%bd%e6%96%b0%e5%9f%ba%e5%bb%ba%e7%ab%9e%e4%ba%89%e5%8a%9b%e6%’

According to the calculation results of the relative progress of all cities, the higher the *C*(*s*_*i*_), the higher the degree of digital transformation of the manufacturing industry.

The article "Digital transformation, industrial structure change, and economic growth motivation: An empirical analysis based on manufacturing industry in Yangtze River Delta" was retracted in 2025. Reasons: unreliable results or conclusions; concerns about the peer review; concerns about the authorship; concerns about the article.

### 3.8. Evaluation result analysis

The scores of the digital transformation degree of the manufacturing industry in 25 cities in the Yangtze River Delta region are ranked in ascending order (Fig 1).

**Fig 1:** Comprehensive evaluation results of digital transformation degree of the manufacturing industry in the Yangtze River Delta region.

As shown in Fig 1, Shanghai, Hangzhou, Nanjing, Nantong, and Wuxi rank among the top five in the Yangtze River Delta region in terms of the degree of digital transformation of the manufacturing industry. These regions should further play an exemplary role in achieving the coordinated development of the manufacturing industry in the Yangtze River Delta. Suqian, Quzhou, Lianyungang, Zhoushan, and Lishui rank in the bottom five in the ranking of the degree of digital transformation of the manufacturing industry in the Yangtze River Delta region, and the digital level of the manufacturing industry in these regions should be further improved.

## 4. Empirical analysis

Using Feder model to construct the two-sector model. Suppose that the economy consists of traditional sectors and digital sectors, and the output of the digital sector has an impact on the output of the traditional sector. The production function of the traditional sector is *T = T* (*K*_*T*_,*L*_*T*_,*D)*, and the production function of the digital sector is *D = D*(*K*_*D*_,*L*_*D*_). Among them, *K*_*T*_ and *K*_*D*_ are capital investments in traditional and digital sectors, *L*_*T*_ and *L*_*D*_ are labor investments in traditional and digital sectors, respectively. The total input is *K = K*_*T*_*+K*_*D*_, *L = L*_*T*_*+L*_*D*_, and the total output of the economy is *Y = T+D*. The output of the digital sector enters the production function of the traditional sector and affects the output level of the traditional sector, so the econometric model is further constructed.

### 4.1 Model

#### 4.1.1 Baseline regression model

Building a benchmark regression model to test the overall effect of manufacturing digitalization on economic growth:

$$Growth_{it}=\alpha_{0}+\beta_{0}DOM_{it}+\gamma_{0}Z_{it}+\mu_{it}$$

Where *i* denotes province and *t* denotes period. *Growth*_*it*_ represents the level of economic growth, is the explained variable; *DOM*_*it*_ represents the level of digital transformation of the manufacturing industry, which is the core explanatory variable; *Z*_*it*_ represents the set of control variables. *α* is a constant term, *μ*_*it*_ is a random disturbance term.

The article "Digital transformation, industrial structure change, and economic growth motivation: An empirical analysis based on manufacturing industry in Yangtze River Delta" was retracted in 2025. Reasons: unreliable results or conclusions; concerns about the peer review; concerns about the authorship; concerns about the article.

#### 4.1.2 Mediation model

Constructing multiple mediating effect model to explore the influence of industrial structure on economic growth under the background of digital transformation of the manufacturing industry:

$$RL_{it}=\alpha_{1}+\beta_{1}DOM_{it}+\gamma_{1}Z_{it}+\varepsilon_{it}$$

$$AL_{it}=\alpha_{2}+\beta_{2}DOM_{it}+\gamma_{2}Z_{it}+\varepsilon_{it}$$

$$II_{it}=\alpha_{3}+\beta_{3}DOM_{it}+\gamma_{3}Z_{it}+\varepsilon_{it}$$

$$Length_{it}=\alpha_{4}+\beta_{4}DOM_{it}+\gamma_{4}Z_{it}+\varepsilon_{it}$$

$$Growth_{it}=\alpha_{5}+\beta_{5}DOM_{it}+\rho_{1}RL_{it}+\rho_{2}AL_{it}+\rho_{3}II_{it}+\rho_{4}Length_{it}+\gamma_{5}\sum CV_{it}+\varepsilon_{it}$$

Among them, the direct effect of manufacturing digital transformation on regional economic growth represents *β*_0_. The mediating effect of influencing through the upgrading of industrial institutions is *β*_1_*ρ*_1_, the mediating effect of influencing through the rationalization of industrial structure is *β*_2_*ρ*_2_, the mediating effect of influencing through the integration of industrial structure is *β*_*3*_*ρ*_*3*_, and the mediating effect of influencing through the upgrading of industrial chain is *β*_*4*_*ρ*_*4*_.

### 4.2 Variable setting

#### 4.2.1 Independent variable: Digital transformation of manufacturing (*DOM*)

We evaluate the degree of digital transformation in the manufacturing industry in 25 cities in the Yangtze River Delta region, draws on the results of existing research on the development of the manufacturing industry and digital transformation, and uses the Pythagoras-TOPSIS method to analyze the degree of digital transformation of manufacturing industry from three dimensions: dynamic capability, platform construction, and organizational system. The evaluation index system of the degree of digital transformation in the manufacturing industry is shown in Table 1. The measurement of index weight is determined by the entropy weight method.

#### 4.2.2 Dependent variable: Economic growth (*Growth*)

Measured by the per capita real GDP data of each city, with 2000 as the base period, the per capita GDP index of the China Statistical Yearbook over the years is calculated.

#### 4.2.3 Mediating variable

Rationalization level of industrial structure (*RI*): reflect the process of industrial structure transformation, pay attention to the coordination degree of industrial development, and realize the rationality of industrial structure development. Using the Theil index to measure production regarding Wu et al.[81], Theil [82].


$$RI=\sum_{i=1}^{n}\frac{Y_{i}}{Y}\ln(\frac{Y_{i}}{L_{i}}/\frac{Y}{L})=\sum_{i=1}^{n}\frac{Y_{i}}{Y}\ln(\frac{Y_{i}}{Y}/\frac{L_{i}}{L})$$

*Yi/Y* and *Li/L* represent the ratio of the total output value of the primary, secondary and tertiary industries to the total regional output value, and the ratio of the total number of labor practitioners in the primary, secondary and tertiary industries to the total number of local practitioners, respectively.

The article "Digital transformation, industrial structure change, and economic growth motivation: An empirical analysis based on manufacturing industry in Yangtze River Delta" was retracted in 2025. Reasons: unreliable results or conclusions; concerns about the peer review; concerns about the authorship; concerns about the article.

The advanced level of industrial structure (*AL*): from the overall consideration of the upgrading of the overall industrial structure, embodied in the increase of product added value and the optimization of the industrial structure of each department. Its measurement method is mainly through sorting the added value of the three industries, to realize the transformation of the industrial structure development of ’ one, two, three ’ into the industrial structure form of ’ three, two, one ’, that is, the industrial structure advanced index, drawing on the practice of Xuan and Peng [83], Fu Linghui [84], etc, we first use the ratio of the added value of the three industries to the regional GDP as the three coordinates of the spatial coordinate system to form a three-dimensional vector, $X_{0}=(x_{1,0},x_{2,0},x_{3,0})$. Then, the industries are arranged from low level to high level, which are expressed as vectors *X*_1_ = (1,0,0), *X*_2_ = (0,1,0), *X*_3_ = (0,1,1), respectively. Calculate the angles between *X*_*0*_ and *X*_*1*_, *X*_*0*_ and *X*_*2*_, *X*_*0*_ and *X*_*3*_, denoted by *θ*_*1*_, *θ*_*2*_, *θ*_*3*_.


$$\theta_{j}=\arccos[\frac{\sum_{i=1}^{3}\left(x_{i,j}x_{i,0}\right)}{\sqrt{\sum_{i=1}^{3}x_{i,j}^{2}}\sqrt{\sum_{i=1}^{3}x_{i,0}^{2}}}],j=1,2,3$$

After calculating the angle, the index of industrial structure upgrading is measured as follows:


$$AL=\sum_{k=1}^{3}\sum_{j=1}^{k}\theta_{j}$$

The larger the value of *AL*, the higher the industrial structure advanced index.

Industrial integration (*II*): Considering the impact of digital transformation on industrial integration, the industrial integration of the information industry and manufacturing industry is analyzed. The input-output principle can be considered from two aspects: input and output. According to the definition of the degree of integration, the input and output between industries are fully considered when measuring the degree of industrial integration, and the degree of industrial integration is measured by the ratio of the information industry input to the total output of the information industry input to the total output of the sub-industry *i*.

The article "Digital transformation, industrial structure change, and economic growth motivation: An empirical analysis based on manufacturing industry in Yangtze River Delta" was retracted in 2025. Reasons: unreliable results or conclusions; concerns about the peer review; concerns about the authorship; concerns about the article.

The length of the industrial chain (*length*_*1i*_): referring to the method of Jeong et al. [85], the upstream degree of the industry is calculated according to the input-output table, and then the relative position of the subdivided industries in the industrial chain is measured. In the process of model construction, we consider a closed economy formed by *N* industries without import and export. For each industry *i (i =* 1,…,*n*), the total output value is the sum of the final consumption *F* of the industry and the intermediate inputs *Z*_*i*_ of other industries, as follows:

$$Y_{i}^{1}=F_{i}+Z_{i}=F_{i}+\sum_{j=1}^{n}a_{ij}Y_{j}^{1}$$

$$a_{ij}=Z_{ij}/Y_{j}^{1}$$

In the formula, *a*_*ij*_ denotes the direct consumption coefficient, and *Z*_*ij*_ denotes the intermediate input of industry *i* required for the output of industry *j*. Measure the length of the 29 manufacturing sub-sector *i* from the final demand, that is, the industrial chain length of industry *i*:

$$length_{1i}=1\times \frac{F_{i}}{Y_{i}^{1}}+2\times \frac{\sum_{j=1}^{n}a_{ij}F_{j}}{Y_{i}^{1}}+3\times \frac{\sum_{j=1}^{n}a_{ik}a_{kj}F_{j}}{Y_{i}^{1}}+4\times \frac{\sum_{j=1}^{n}a_{il}a_{lk}a_{kj}F_{j}}{Y_{i}^{1}}+\ldots +29\times \frac{\sum_{j=1}^{n}a_{il}....a_{kj}F_{j}}{Y_{i}^{1}}$$

*length*_*1i*_≥1, the greater the value, the longer the industrial chain. Assuming that the direct consumption coefficient remains unchanged for a certain period, the direct consumption coefficient is calculated by using the 2012 input-output table as the direct consumption coefficient from 2010 to 2014. The direct consumption coefficient from 2015 to 2020 is calculated by using the 2017 input-output table.

#### 4.2.4 Control variables

Selecting human capital stock, government size, total fixed assets, and enterprise size as control variables, it is possible to achieve cumulative value-added benefits and economic growth by expanding the scale of use.

*4*.*2*.*4*.*1*. *Human capital stock* (HCS)

Using the ratio of employment to the total population of the region to measure, employment data from the ’China City Statistical Yearbook’ in the secondary industry employment.

*4*.*2*.*4*.*2*.*Government size* (CS)

Measured by the proportion of regional government expenditure to GDP. The small size of the government will lead to an insufficient supply of public goods, especially insufficient investment in digital infrastructure, which may adversely affect long-term economic growth.

*4*.*2*.*4*.*3*. *Total fixed assets* (TFA)

It is expressed by the total fixed assets of manufacturing enterprises. The total fixed assets are calculated according to the following formula:

$$K_{T}=K_{0}+\sum_{t=1}^{T}\Delta K_{i}/P_{t}$$

*K*_*T*_ is the total fixed assets of the year *T*; *K*_*0*_ is the annual average balance of net fixed assets in 2000, is the increase in net fixed assets in year *t*, and *P*_*t*_ is the fixed asset investment price index in year *t* converted with 2000 as the base period.

*4*.*2*.*4*.*4*. *Enterprise size* (ES). In the ’’14th Five-Year’’ intelligent manufacturing development plan, put forward the goal of a digital network of manufacturing enterprises above the designated size. Therefore, enterprise scale plays an important role in the digital transformation of manufacturing industry. At the same time, studies have pointed out the relationship between the growth of the number of enterprises and economic growth. Therefore, taking the scale of enterprises as the control variable, which is measured by the logarithm of the total assets of the enterprise.

The article "Digital transformation, industrial structure change, and economic growth motivation: An empirical analysis based on manufacturing industry in Yangtze River Delta" was retracted in 2025. Reasons: unreliable results or conclusions; concerns about the peer review; concerns about the authorship; concerns about the article.

## 5. Results

The data come from China Industry Economy Statistical Yearbook, China City Statistical Yearbook, China Labor Statistical Yearbook, China Economic Census Yearbook, the National Research Network database, the National Bureau of Statistics, the China Statistical Yearbook. All indicators are based on current year price data as a constant price. The total fixed assets data are standardized. Relevant specific data sets can be accessed through direct hyperlinks. Others will be able to access or request this data in the same way as the author, who does not have any special access or request privileges that others will not have.

China Industry Economy Statistical Yearbook:

https://www.yearbookchina.com/naviBooklist-n3021030901-1.html

China City Statistical Yearbook from Zhejiang and Anhui provinces and Shanghai Municipal Bureau of Statistics website:

https://tjj.sh.gov.cn/tjnj/

http://tjj.zj.gov.cn/col/col1525563/index.html

http://tjj.ah.gov.cn/ssah/qwfbjd/tjnj/index.html

China Labor Statistical Yearbook:

http://www.mohrss.gov.cn/

China Economic Census Yearbook:

China. China Economic Census Yearbook. 2013 Volume I [M]. China Statistical Press, 2013.

China. China Economic Census Yearbook. 2018 Volume I [M]. China Statistical Press, 2018.

National Research Network database

http://www.drcnet.com.cn/www/int/

the National Bureau of Statistics:

http://www.stats.gov.cn/

the China Statistical Yearbook:

http://www.shujuku.org/

The descriptive statistical results are shown in Table 2.

**Table 2:** Variables descriptive statistics.

Variable	Observations	Mean	Standard deviation	Minimum	Median	Maximum
*DOM*	352	0.6167	0.1482	0.4219	0.6345	0.8894
*Growth*	352	1.1684	0.0681	1.0034	1.1574	1.2798
*RI*	352	0.8704	0.4003	0.3871	0.7561	0.9984
*AL*	352	0.5542	0.1137	0.4264	0.5741	0.7897
*II*	352	0.1567	0.0641	0.0962	0.1845	0.2553
*Length*	352	1.2354	0.3002	0.8571	1.2641	1.6035
*HCS*	352	0.5624	0.2567	0.2031	0.6214	0.9024
*CS*	352	0.1035	0.1958	0.0525	0.1004	0.1695
*TFA*	352	0.5561	0.2567	0.0000	0.5984	1.0000
*ES*	352	0.3871	0.0891	0.2655	0.3841	0.5062

The article "Digital transformation, industrial structure change, and economic growth motivation: An empirical analysis based on manufacturing industry in Yangtze River Delta" was retracted in 2025. Reasons: unreliable results or conclusions; concerns about the peer review; concerns about the authorship; concerns about the article.

### 5.1. Multicollinearity test of variables

Use tolerance and variance inflation factors to test multicollinearity between variables. The tolerance of all variables is above 0.5 level, the tolerance is greater than 0.1, and the variance expansion factor is less than 2. The variance inflation factor did not exceed the highest standard for judging the multicollinearity of variables (Table 3).

**Table 3:** Multicollinearity test results of regression model variables.

Variables	Non-standardized coefficient		Standardized		Sig.	Colinearity statistics	
	Coefficient	Standard error	Coefficient	Standard error		Tolerance	VIF
*DOM*	0.8057	0.2420	0.0679	1.5419	0.0000	0.7379	1.2813
*AL*	0.9264	0.2243	0.2405	0.8133	0.0000	0.6450	1.5642
*RI*	0.7939	0.3167	0.0183	0.4342	0.0000	0.5908	1.1061
*II*	0.6835	0.1948	0.1032	0.5831	0.0000	0.6231	1.0293
*length*_*1i*_	0.5858	0.1055	0.1165	0.3825	0.0000	0.5968	0.9845

### 5.2. Benchmark model regression results

The individual fixed effect model is selected for parameter estimation, and the stepwise regression method is used to empirically test the impact of the digital transformation of the manufacturing industry on economic growth (Table 4). Model (1) only adds explanatory variables for regression. The results show that manufacturing digitization has a significant positive impact on economic growth. Model (2) to Model (5) gradually add control variables (*HCS*, *CS*, *TFA*, *ES*). With the addition of control variables one by one, the explanatory power of the model is enhanced and effective.

**Table 4:** Regression results of panel fixed effect of digital transformation of manufacturing industry on economic growth.

Variables	(1)	(2)	(3)	(4)	(5)
*DOM*	2.9157* (0.1841)	2.8350*** (0.2050)	2.8445*** (0.2157)	0.7793** (0.1410)	0.7793*** (0.1410)
*HCS*	—	0.1926 (0.1852)	0.1958 (0.1867)	0.3137* (0.0770)	0.0656 (0.1113)
*CS*	—	—	-0.1838* (1.2860)	0.1733** (0.0657)	0.4022 (0.7392)
*TFA*	—	—	—	0.1646** (0.0328)	0.3900*** (0.0139)
*ES*	—	—	—	—	0.1311*** (0.0178)
*CONT*	1.0968*** (0.1368)	1.0755*** (0.1504)	0.9077*** (0.1512)	0.4633 (0.4778)	0.9548 (0.1178)
Individual Fixed effect	Control	Control	Control	Control	Control
R^2^	0.3167	0.3276	0.3277	0.7485	0.7914
*Adj*.R^2^	0.3084	0.3243	0.3226	0.7446	0.7810
Number of observations	352	352	352	352	352

Note: ***, **, and * are significant at the 1%, 5%, and 10% levels, respectively, and the robust standard error is in parentheses, the same below.

The article "Digital transformation, industrial structure change, and economic growth motivation: An empirical analysis based on manufacturing industry in Yangtze River Delta" was retracted in 2025. Reasons: unreliable results or conclusions; concerns about the peer review; concerns about the authorship; concerns about the article.

From the perspective of core explanatory variables, the digital transformation of the manufacturing industry has a significant positive impact on economic growth, which verifies hypothesis 2. A significant positive relationship between the digital transformation of the manufacturing industry and the technical effect. In the process of gradually adding control variables, the positive effect of the digital transformation of the manufacturing industry on economic growth shows a downward trend, indicating that there may be heterogeneous factors in the effect of the digital transformation of the manufacturing industry on economic growth. Aiming at the actual effect of manufacturing digitization promoting industrial structure leading to economic growth in hypothesis 3, the specific manifestation of the relationship between the ’ manufacturing digitization transformation-industrial structure-economic growth ’ of manufacturing enterprises is presented through path relationship. Firstly, the direct effect of industrial structure on economic growth is tested (Table 5).

**Table 5:** Test results of the direct effect of industrial structure on economic growth.

Variables	Dependent variable: Growth				
	(6)	(7)	(8)	(9)	(10)
*DOM*	1.0256*** (0.1670)	0.7748*** (0.1369)	0.1312* (0.0756)	0.7072*** (0.1213)	0.2651*** (0.0915)
*HCS*	0.0900 (0.1123)	0.1269* (0.103)	0.0436 (0.1963)	0.1719* (0.0974)	0.1505 (0.1935)
*CS*	0.4820 (0.7332)	-0.0905 (0.7250)	-0.0978* (0.7123)	2.4705*** (0.1213)	1.5559*** (0.6328)
*TFA*	0.3873***(0.0138)	0.3455*** (0.0164)	0.3128* (0.0188)	0.2680*** (0.0162)	0.1716*** (0.0199)
*ES*	0.1311***(0.0178)	0.1641** (0.0539)	0.1327** (0.0482)	0.1594*** (0.0384)	0.1657* (0.0968)
*AL*	0.2212***(0.0820)	—	—	—	0.0383* (0.0190)
*RI*	—	0.2974*** (0.0629)	—	—	0.1675** (0.0534)
*II*	—	—	0.0518*** (0.0090)	—	0.0528*** (0.0008)
*length*_*1i*_	—	—	—	0.2684*** (0.0241)	0.2527** (0.0233)
*F*	269.48	283.96	294.44	381.52	283.68
*R* ^*2*^	0.7957	0.8041	0.8097	0.8465	0.8687
*Adjusted-R* ^2^	0.7927	0.8012	0.8070	0.8442	0.8656
Number of observations	352	352	352	352	352

Our research further supplements and extends the research results of Nambisan et al., Yoo and Yi [86, 87]. From the perspective of conceptual integration, we study the principle that digital technology, digital platform and digital infrastructure transform organizational and social relations through value creation and value capture. Yoo and Yi reviewed the research on digital transformation and economic growth through systematic literature review, and explained the connection between digitization and social system from a comprehensive framework. They believe that digital innovation has led to changes in the industrial structure, thereby reducing costs [87]. Our research further derives the path of ’ manufacturing digital transformation-industrial structure-economic growth ’ from the mechanism of manufacturing digitization, which explains how to promote the co-evolution of technology, economy, society and policy sectors from the whole.

The article "Digital transformation, industrial structure change, and economic growth motivation: An empirical analysis based on manufacturing industry in Yangtze River Delta" was retracted in 2025. Reasons: unreliable results or conclusions; concerns about the peer review; concerns about the authorship; concerns about the article.

### 5.3. The mediating effect test of industrial structure

Whether the digital transformation of the manufacturing industry has an impact on economic growth through the industrial structure, further application of step-by-step test method to test the impact of digital manufacturing industry on the industrial structure, and analysis of the intermediary effect of industrial structure variables. Therefore, first of all, the advanced industrial structure as the dependent variable, the human capital stock, government size, total fixed assets, and firm size in the regression model 5, the results show that the control variables can pass the significance test. Further digital transformation of manufacturing into the model, the results show that digital transformation of manufacturing can positively affect the upgrading of industrial structure. The second step is to continue to use the rationalization of industrial structure, the integration of industrial structure, and the length of the industrial chain as dependent variables, and also incorporate control variables into the regression model to analyze whether the digital transformation of the manufacturing industry can have a different impact on industrial structure. The regression coefficients of manufacturing digitalization on industrial structure all pass the significance test (Table 6). In the third step, taking economic growth as the dependent variable, the industrial structure upgrading index, industrial structure rationalization, industrial structure integration and industrial chain length variables, four control variables, and manufacturing digital transformation variables are included in the regression model to analyze the mediating role of different variables. The results of model (19) and model (20) show that when the independent variables and intermediary variables of the digital transformation of the manufacturing industry are included in the regression model at the same time, the coefficient of industrial structure upgrading is 0.1485 (p<0.05), the coefficient of industrial structure rationalization is 0.1574 (p<0.01), the coefficient of industrial structure integration is 0.1095 (p<0.01), and the coefficient of industrial chain length is 0.0748 (p<0.05). The coefficient of manufacturing digital transformation decreased from 0.1536 (p<0.01) to 0.1234 (p<0.01). Therefore, the industrial structure variable plays a partial mediating role in the relationship between manufacturing digital transformation and economic growth. Among them, the advanced industrial structure and the length of the industrial chain coefficient are larger, and the positive impact on economic growth is higher.

The article "Digital transformation, industrial structure change, and economic growth motivation: An empirical analysis based on manufacturing industry in Yangtze River Delta" was retracted in 2025. Reasons: unreliable results or conclusions; concerns about the peer review; concerns about the authorship; concerns about the article.

**Table 6:** Measurement results of mediating effect.

Variables	*AL*		*RI*		*II*		*length*_*1i*_		*Growth*	
	(11)	(12)	(13)	(14)	(15)	(16)	(17)	(18)	(19)	(20)
*HCS*	0.1296**	0.1414**	0.1511**	0.1412**	0.1203*	0.0983*	0.1095**	0.1854*	0.1135**	0.1093**
*CS*	0.1416**	0.1461**	0.2637**	0.1107**	0.1061*	0.1615*	0.0818**	0.0957**	0.1253**	0.1137*
*TFA*	0.1047*	0.2110*	0.2266**	0.1408*	0.0743**	0.0962**	0.1135***	0.1024*	0.1074*	0.1142**
*ES*	0.1605**	0.1138*	0.1593***	0.2011***	0.0945***	0.1025**	0.1501***	0.1242*	0.1033*	0.1038**
*DOM*	—	0.2071***	—	0.2010***	—	0.1014**	—	0.0936***	0.1536***	0.1234***
*RI*	—	—	—	—	—	—	—	—	—	0.2485**
*AL*	—	—	—	—	—	—	—	—	—	0.0574***
*II*	—	—	—	—	—	—	—	—	—	0.0095***
*Length*	—	—	—	—	—	—	—	—	—	0.2148**
*F*	0.184	36.275	58.326	0.113	42.264	103.425	218.211	210.583	205.328	203.735
*R* ^*2*^	0.013	0.484	0.158	0.415	0.217	0.474	0.217	0.593	0.537	0.602
*Adj*.*R*^*2*^	0.011	0.481	0.152	0.409	0.212	0.472	0.213	0.589	0.532	0.599
Number of observations	352	352	352	352	352	352	352	352	352	352

The results of the analysis of the mediating effect of the industrial structure show that there are four transmission paths for digital transformation to affect economic growth, which demonstrates the important judgment that digital transformation affects economic growth through the industrial structure in the field of manufacturing production, and further shows the important role of digital transformation of manufacturing enterprises in promoting the upgrading of industrial structure and extending the industrial chain. The mediating effect of the industrial structure reveals the ’result attribute’ and ’path attribute’ of digital transformation of manufacturing affecting economic growth.

Our study further complements the results of Shi [88] and Zhang [89]. They believe that industrial structure optimization is an important explanatory variable of economic growth. However, they only explained its role in economic growth from the perspective of industrial structure evolution. Our empirical results show that the digital transformation of manufacturing industry is the antecedent of industrial structure upgrading, which promotes economic growth through the mediating effect of industrial structure upgrading, rationalization, industrial integration and optimization. Therefore, our research is conducive to a comprehensive understanding of the role of industrial upgrading in economic growth and is of great significance for China ’s economic development.

The article "Digital transformation, industrial structure change, and economic growth motivation: An empirical analysis based on manufacturing industry in Yangtze River Delta" was retracted in 2025. Reasons: unreliable results or conclusions; concerns about the peer review; concerns about the authorship; concerns about the article.

Considering the adequacy of the selected samples, Bootstrap is set to 1000 times of repeated sampling. SPSS macro PROCESS and Bootstrap method are further applied to test the differences of four mediating effects of industrial structure upgrading, industrial structure rationalization, industrial structure integration, and industrial chain length (Table 7).

**Table 7:** Difference of mediating effect of industrial structure.

Mediation model	Manufacturing Digital Transformation—Economic Growth				
Direct effect	Effect	SE	*t*	*p*	LLCI, ULCI
	0.0964	0.0362	1.2854	0.0123	[0.0648, 0.2028]
Indirect effect: *AL*	Effect		Boot SE		Boot LLCI, Boot ULCI
	0.0866		0.0753		[0.0684, 0.3655]
Direct effect	Effect	SE	*t*	*p*	LLCI, ULCI
	0.1226	0.1052	1.7426	0.0371	[0.1157, 0.3422]
Indirect effect: *RI*	Effect		Boot SE		Boot LLCI, Boot ULCI
	0.0826		0.0374		[0.0462, 0.2003]
Direct effect	Effect	SE	*t*	*p*	LLCI, ULCI
	0.1011	0.0214	1.2354	0.0125	[0.0783, 0.2068]
Indirect effect: *II*	Effect		Boot SE		Boot LLCI, Boot ULCI
	0.0955		0.0529		[0.0546, 0.2015]
Direct effect	Effect	SE	*t*	*p*	LLCI, ULCI
	0.1417	0.0652	1.6437	0.0286	[0.0916, 0.2768]
Indirect effect: *length*_*1i*_	Effect		Boot SE		Boot LLCI, Boot ULCI
	0.1055		0.0973		[0.0643, 0.1645]
Total	0.5184		0.1004		[0.1486, 0.6542]
*AL*	0.1732		0.0721		[0.0427, 0.2817]
*RI*	0.0658		0.0664		[0.0593, 0.3171]
*II*	0.0960		0.1216		[0.0827, 0.1713]
*length*_*1i*_	0.1834		0.1037		[0.0647, 0.2139]

The results show that when the industrial structure upgrading is examined separately, the confidence interval of the direct effect is [0.0648,0.2028], and the confidence interval of the indirect effect is [0.0684,0.3655], both of which do not contain zero values. Therefore, the upgrading of the industrial structure plays an intermediary role in the relationship between digital transformation and economic growth. When the rationalization of industrial structure is investigated separately, the confidence interval of direct effect is [0.1157,0.3422], and the confidence interval of indirect effect is [0.0462,0.2003], both of which do not contain zero value. Therefore, the technical effect plays an intermediary role in the relationship between digital transformation and economic growth; when the degree of industrial integration is examined separately, the confidence interval of the direct effect is [0.0783,0.2068], and the confidence interval of the indirect effect is [0.0546,0.2015], both of which do not contain zero values. Therefore, industrial integration has a mediating effect on the impact of digital transformation on economic growth; when the length of the industrial chain is examined separately, the confidence interval of the direct effect is [0.0916,0.2768], and the confidence interval of the indirect effect is [0.0643,0.1645], both of which do not contain zero values. Therefore, digital transformation can promote economic growth by extending the length of the industrial chain.

The article "Digital transformation, industrial structure change, and economic growth motivation: An empirical analysis based on manufacturing industry in Yangtze River Delta" was retracted in 2025. Reasons: unreliable results or conclusions; concerns about the peer review; concerns about the authorship; concerns about the article.

The development of digital economy can promote the rationalization and upgrading of industrial structure, so as to realize the transformation and upgrading of industrial structure. Our research further expounds the profound influence of industrial integration, complements and verifies the research results of Li [90] and Chen [91].

When comprehensively analyzing the multiple mediating effects of industrial structure, the confidence interval of the overall indirect effect of industrial structure is [0.1486,0.6542], excluding zero value; The indirect effects of an industrial structure optimization, industrial structure rationalization, industrial structure integration, and industrial chain length are 0.1732, 0.0658, 0.0960 and 0.1834 respectively. Therefore, under the condition of existing digital technology and platform construction of manufacturing enterprises, the intermediary role of industrial structure upgrading and industrial chain integration is the dominant direction for the industrial structure to play an intermediary role.

### 5.4. Robustness test

In the process of digital transformation of manufacturing industry promoting urban economic growth, digital transformation and economic development are two key contents in the process of urban construction. There may be a certain linkage between digital transformation of manufacturing industry and urban economic growth. It is difficult to avoid maintaining absolute independence and exogenousness, and they may be affected by urban economic development in the process of considering the digital transformation of urban manufacturing. This correlation may lead to the endogenous problem of reverse causality when studying the digital transformation of manufacturing industry and urban economic growth, resulting in the bias of parameter estimation results. At the same time, if the missing variables that affect the digital transformation of manufacturing industry and urban economic growth cannot be controlled, the influence between the explanatory variables and the explained variables will not be identified. Therefore, it is necessary to find variables that are closely related to the digital transformation of urban manufacturing, but are not related to missing variables, which can better identify the causal impact.

The article "Digital transformation, industrial structure change, and economic growth motivation: An empirical analysis based on manufacturing industry in Yangtze River Delta" was retracted in 2025. Reasons: unreliable results or conclusions; concerns about the peer review; concerns about the authorship; concerns about the article.

Appropriate instrumental variables (IV) are used to control endogeneity in order to obtain more reliable empirical analysis. Appropriate instrumental variables are highly correlated with endogenous variables, ensuring sufficient exogeneity, that is, instrumental variables only affect the explanatory variables through endogenous variables. Digital infrastructure construction is the core base of digital development and transformation of manufacturing industry, and the key to ensure the effective progress of digital manufacturing industry.

Logically, the digital transformation of urban manufacturing industry will be directly affected by digital infrastructure investment, and the correlation assumption between effective instrumental variables and endogenous variables can be satisfied. Second, digital infrastructure investment has more natural exogenous characteristics, which well satisfies the exogenous assumption of effective instrumental variables. Therefore, we use the logarithm of digital infrastructure investment as an instrumental variable. The results of IV-GMM are shown in Table 8.

**Table 8:** The generalized moment estimation results of manufacturing digital transformation on economic growth.

*Variables*	*AL*	*RI*	*II*	*length*_*1i*_	*Growth*
*DR*	0.7642*** (0.2357)	0.2594** (0.0951)	0.1698*** (0.0367)	1.0357*** (0.0294)	0.3065** (0.0564)
*AL*	—	—	—	—	0.1894*** (0.0451)
*RI*	—	—	—	—	0.6254*** (0.0897)
*II*	—	—	—	—	0.1583** (0.0621)
*length*_*1i*_	—	—	—	—	0.9572*** (0.2684)
Control variable	Control	Control	Control	Control	Control
Observations	352	352	352	352	352
R-squared	0.3358	0.3694	0.4851	0.4937	0.7051
Wald-F stat	62.348	69.881	75.648	78.852	152.348
p-value	0.3218	0.3365	0.2984	0.2851	0.1681

Note: In parentheses are t statistical test values, *means p < 0.1, ** means p < 0.05, *** means p < 0.01; wald-Fstat > 1.96 indicates that the instrumental variable is not a weak instrumental variable; p > 0.05, accept the null hypothesis, indicating that the instrumental variable is an exogenous variable.

The results show that all instrumental variables are exogenous. In the first stage of regression, the coefficients of instrumental variables are significantly not equal to zero, and the sign direction is consistent with expectations. In the second stage of regression, the significance and symbolic direction of the core explanatory variables are consistent with the benchmark regression results. Therefore, after considering the endogenous problem, the digital transformation and development of the manufacturing industry can still significantly promote economic growth.

## 6. Discussion

On the one hand, the direct effect of the digital transformation of the manufacturing industry on economic growth reflects the management characteristics of the economic growth effect of enterprise digital technology development, dynamic capability construction, platform, and system construction. On the other hand, the indirect effect of digital transformation of the manufacturing industry on economic growth reflects the correlation characteristics of economic growth effect through the industrial structure in the process of developing digital technology in the whole process. This shows that manufacturing enterprises should pay attention to the influencing factors of production management, organizational system, and industrial digital development in the process of digital transformation.

The article "Digital transformation, industrial structure change, and economic growth motivation: An empirical analysis based on manufacturing industry in Yangtze River Delta" was retracted in 2025. Reasons: unreliable results or conclusions; concerns about the peer review; concerns about the authorship; concerns about the article.

The empirical analysis results show that digital transformation promotes the transformation and upgrading of the industrial structure of the manufacturing industry. The higher the degree of digital transformation of the manufacturing industry through information interconnection and technology sharing among enterprises, the greater the positive impact on economic growth. With the increasing degree of digital transformation of manufacturing enterprises, the application of digital technology and input costs will be reduced. Economic growth was promoted by increasing synergy between sectors. The mediating effect test shows the indirect mechanism of manufacturing digitization positively affects economic growth. Industrial structure upgrading and industrial chain integration are two important paths in the process of digital transformation of the manufacturing industry to promote economic growth.

Comprehensive analysis of the impact of digital transformation of the manufacturing industry on economic growth through the industrial structure from the dimensions of result attribute and path attribute is the key to comprehensively analyzing the law and influence degree of digital transformation of the manufacturing industry. Therefore, we propose the following management implications:

(1) Improve the dynamic capability of manufacturing enterprises. Relying on digital information technology, at the enterprise level, industrial Internet, big data, cloud networks, artificial intelligence, and other digital technologies are widely used to improve the flexible production capacity of enterprises. (2) Promote the establishment of information statistics and analysis platforms. Establish an enterprise product information database to ensure the smooth exchange of information between the various management departments, and production management body. (3) Improve the organizational digitization system. Using big data to overcome the organizational segmentation of enterprise space and time. (4) Promote the optimization of industrial structure. At the government level, guide the digital transformation of manufacturing industry development.

The article "Digital transformation, industrial structure change, and economic growth motivation: An empirical analysis based on manufacturing industry in Yangtze River Delta" was retracted in 2025. Reasons: unreliable results or conclusions; concerns about the peer review; concerns about the authorship; concerns about the article.

### 6.1. Limitation of the study and future recommendation

This study has certain limitations and can provide direction for future research. First of all, the integration of digital technology and manufacturing production sectors will help optimize and adjust the industrial structure in the long run. Digitization of manufacturing industry can improve the quality and efficiency of the supply side, promote the networking, openness and synergy of the innovation system, change the direction of market investment, promote consumption upgrading, form new driving forces for economic development and promote high-quality economic development. Future research can consider supplementing theories, combining other theoretical perspectives such as market, investment and consumption and industrial upgrading, and deeply exploring the internal mechanism of digital transformation of manufacturing industry affecting industrial upgrading and promoting economic development. Second, on August 17,2013, the State Council of China issued the " Broadband China " strategy implementation plan, which raised the " Broadband Strategy " from a departmental action to a national strategy and became the " central node " and " transmission link " of the spatial network of the modern economic system. The research sample time of this paper is 2014–2020, without considering the possible impact of the ’ Broadband China ’ strategy. In the future, the impact of the strategy on economic growth can be further considered. Third, our research only considers the impact of digital transformation of manufacturing industry on economic growth. However, the management mode, organizational structure, enterprise scale and innovation ability of manufacturing enterprises themselves may have an impact in this process. In this regard, in the future, micro variables at the enterprise level can be further increased to determine whether the digital transformation of the manufacturing industry is affected by the enterprise level, so as to improve the generalization of the research conclusions.

## 7. Conclusions

We construct an evaluation index system for the degree of digital transformation of the manufacturing industry and study the relationship between manufacturing digitization, industrial structure, and economic growth momentum. The results show that: (1) The digital transformation of the manufacturing industry has a significant positive effect on economic growth. The sharing of knowledge, resources, and technology across organizations through digital platforms further strengthens the information exchange between enterprises, which helps manufacturing enterprises to grasp the production rules, thus reducing the uncertainty faced in the production process and achieving economic growth. (2) Digital transformation improves the rationalization level of industrial structure upgrading, effectively extends the length of the industrial chain, and the integration of manufacturing and information industry reduces the uncertainty of the production process. (3) Manufacturing digitalization forms a new driving force for economic growth by promoting the upgrading of industrial structure. Among them, the positive effect of industrial structure upgrading and industrial chain integration on economic growth becomes more and more obvious with the deepening of manufacturing digitalization.
